The article "Analysis of China’s carbon market price fluctuation and international carbon credit financing mechanism using random forest model" was retracted in 2025. Reasons: concerns about the results or conclusions; concerns about the peer review; concerns about the authorship.

# Analysis of China’s carbon market price fluctuation and international carbon credit financing mechanism using random forest model

**DOI:** 10.1371/journal.pone.0294269

**Published:** 2024-03-07

**Authors:** Cuiling Song

**Affiliations:** School of Financial Technology, Suzhou Industrial Park Institute of Services Outsourcing, Jiangsu, Suzhou City, China; University of Galway, Ireland / Anhui University of Finance and Economics, CHINA

## Abstract

This study aims to investigate the price changes in the carbon trading market and the development of international carbon credits in-depth. To achieve this goal, operational principles of the international carbon credit financing mechanism are considered, and time series models were employed to forecast carbon trading prices. Specifically, an ARIMA(1,1,1)-GARCH(1,1) model, which combines the Generalized Autoregressive Conditional Heteroskedasticity (GARCH) and Autoregressive Integrated Moving Average (ARIMA) models, is established. Additionally, a multivariate dynamic regression Autoregressive Integrated Moving Average with Exogenous Inputs (ARIMAX) model is utilized. In tandem with the modeling, a data index system is developed, encompassing various factors that influence carbon market trading prices. The random forest algorithm is then applied for feature selection, effectively identifying features with high scores and eliminating low-score features. The research findings reveal that the ARIMAX Least Absolute Shrinkage and Selection Operator (LASSO) model exhibits high forecasting accuracy for time series data. The model’s Mean Squared Error, Root Mean Squared Error, and Mean Absolute Error are reported as 0.022, 0.1344, and 0.1543, respectively, approaching zero and surpassing other evaluation models in predictive accuracy. The goodness of fit for the national carbon market price forecasting model is calculated as 0.9567, indicating that the selected features strongly explain the trading prices of the carbon emission rights market. This study introduces innovation by conducting a comprehensive analysis of multi-dimensional data and leveraging the random forest model to explore non-linear relationships among data. This approach offers a novel solution for investigating the complex relationship between the carbon market and the carbon credit financing mechanism.

## 1 Introduction

With the progress of economic development, energy consumption has steadily increased, giving rise to global concerns regarding climate and environmental changes caused by greenhouse gas emissions, particularly carbon dioxide [1–3]. Consequently, carbon dioxide emissions have become a noteworthy production factor for enterprises, now integrated into their cost structure, necessitating a shift in their understanding to acknowledge that fossil energy consumption and carbon dioxide emissions entail additional costs [4–6]. This changing landscape of green consumption and the emerging demand for carbon neutrality across the entire industrial chain has motivated small and medium-sized enterprises to proactively participate in the carbon trading market [7]. In the context of growing global apprehension regarding climate change and carbon emissions, establishing carbon markets and evolving international carbon credit financing mechanisms have emerged as profoundly significant subjects. The carbon trading mechanism has bestowed defined market value upon carbon assets, rendering them potential collateral or mortgage instruments, serving as a credit enhancement measure. This also exemplifies the recognition of carbon emission rights as corporate assets [8]. In the process of financial institutions adjusting social resource allocation and industrial structure, credit products play a pivotal role [9]. As an innovative financial tool, green credit incorporates environmental considerations into traditional credit products offered by commercial banks, enabling the screening of high-energy-consuming and high-polluting enterprises, thereby withholding credit support [10–12]. The resultant carbon credit financing mechanism holds significant potential for China to establish a robust low-carbon development circular green economic system.

The article "Analysis of China’s carbon market price fluctuation and international carbon credit financing mechanism using random forest model" was retracted in 2025. Reasons: concerns about the results or conclusions; concerns about the peer review; concerns about the authorship.

China is currently in the initial stage of establishing a carbon trading market. It is imperative to draw insights from domestic and international experiences while considering the carbon trading prices as a critical connection linkage to fostering the development of a robust carbon trading market in China [13–15]. Ensuring policy system stability and the soundness of laws and regulations is crucial to achieve this scheme. Establishing carbon markets not only enhances enterprises’ carbon emissions management and generates market value for carbon assets. Simultaneously, carbon credit financing mechanisms offer vital financial support for the advancement of China’s low-carbon, circular, and green economic system. However, beyond these benefits, the volatility in carbon market price fluctuations can potentially threaten the market’s effective operation. Therefore, an efficient carbon trading market needs to maintain stable price fluctuations in carbon trading to ensure smooth market operations [16–18]. The stability of carbon trading prices is of paramount importance as volatile transaction prices in the carbon market pose significant financial risks. These risks may impede market capitalization and activity, thus undermining the market’s effectiveness in promoting energy conservation and emission reduction efforts [19]. Consequently, it becomes essential to accurately predict the trend of market price fluctuations and effectively mitigate this risk. In this context, machine learning, known for its exceptional generalization capabilities in price prediction, holds promising applications in the carbon market [20–22]. Prior research has demonstrated the substantial potential of machine learning models in price prediction. Models such as support vector machines and random forests offer viable approaches in terms of prediction accuracy and fitting degree. The random forest model, known for its capacity to model non-linear relationships and handle high-dimensional data, serves as a potent tool for enhancing the accuracy of carbon market price fluctuation predictions.

The article "Analysis of China’s carbon market price fluctuation and international carbon credit financing mechanism using random forest model" was retracted in 2025. Reasons: concerns about the results or conclusions; concerns about the peer review; concerns about the authorship.

This study commences with an examination of the existing state of carbon trading prices and the international carbon credit financial market. In light of China’s dual carbon goals, a suitable international carbon credit financing mechanism is proposed. The study introduces an innovative approach by utilizing a combined time series model. The proposed model demonstrates a high degree of accuracy in predicting the temporal fluctuations of carbon prices. Moreover, the study presents a novel methodology that employs a random forest model to forecast the volatility trends in carbon market prices, followed by comprehensive data analysis. These significant findings provide valuable insights for China to establish a comprehensive carbon trading market and foster the advancement of a sustainable, green, and low-carbon economy. The research innovation hinges on the adoption of the random forest model, a potent machine learning technique for forecasting price fluctuations within the carbon market. This novel approach effectively addresses the constraints associated with conventional statistical models and excels in managing high-dimensional data and non-linear relationships. Consequently, this method offers a fresh avenue for precise carbon market price predictions. This model’s robustness is particularly well-suited for analyzing complex relationships, making it a valuable addition to the research. Moreover, the study’s distinctive contribution lies in the integration and analysis of data from two different domains, namely carbon market price fluctuations and international carbon credit financing mechanisms. This comprehensive approach allows for a thorough investigation of the interaction between these two domains, shedding new light on their interconnected dynamics.

The article "Analysis of China’s carbon market price fluctuation and international carbon credit financing mechanism using random forest model" was retracted in 2025. Reasons: concerns about the results or conclusions; concerns about the peer review; concerns about the authorship.

## 2 Literature review

China’s carbon trading market has been relatively nascent, characterized by an evolving trading mechanism and intricate volatility in carbon prices, influenced by macroeconomic conditions, market environment, and abnormal weather patterns. Given the importance of comprehending the factors that affect carbon trading prices, research in this domain has attracted considerable attention from experts and scholars both domestically and internationally. For instance, Siyal et al. (2021) [23] investigated the impact of carbon market price fluctuations on commercial banks. Hu et al. (2021) [24] explored strategies for cultivating diverse talents in the field of carbon finance. Davoodi et al. (2023) [25] presented a novel hybrid forecasting framework to address the challenges in carbon price prediction, incorporating diverse influencing factors through advanced algorithms. The study introduced a kernel-based optimal extreme learning machine model, which efficiently combines the multi-objective chaotic sine-cosine algorithm optimizer, demonstrating outstanding generalization and stability. Lu et al. (2020) [26] predicted China’s carbon trading volume and price using a machine learning model with an innovative data denoising technique incorporating empirical mode decomposition with adaptive noise to successfully smooth raw data. Hao et al. (2020) [27] proposed a novel hybrid model that integrated feature selection and a multi-objective optimization algorithm for carbon price forecasting, yielding lower average absolute percentage errors compared to other comparative models, with values of 2.4923% and 0.8418%, respectively.

Cai & Ya (2022) [28] utilized a dynamic recursive computation general equilibrium model to analyze the influence of various emission trading schemes on carbon trading price levels. The study’s results reveal that with an increase in carbon emission trading price levels, the decline in the gross domestic product becomes more prominent, indicating a higher sensitivity of the energy industry to carbon emission trading prices in comparison to other industries. In a similar vein, Venmans et al. (2020) [29] conducted a comprehensive review of ex-post empirical assessments that examined the impact of carbon pricing on competitiveness in the power and industrial sectors across the Organization for Economic Co-operation and Development and G20 countries, primarily focusing on the European Union (EU). Most of these assessments did not find statistically significant effects of carbon pricing or energy prices on various dimensions of competitiveness. In addition, Huang & He (2020) [30] proposed a novel combinatorial optimization forecasting method that integrated unstructured data based on factors such as gray correlation analysis, factor analysis, and the Baidu index. This approach utilized both structured and unstructured data as inputs for prediction. Niu et al. (2022) [31] developed a hybrid prediction system integrating error correction and divide-and-conquer strategies to achieve accurate forecasts of carbon price sequences. Their approach involved a data-preprocessing module based on the divide-and-conquer strategy, an optimization module utilizing the multi-objective grasshopper optimization algorithm to enhance prediction performance, and an error correction module in predicting error sequences and adjusting model results accordingly.

The article "Analysis of China’s carbon market price fluctuation and international carbon credit financing mechanism using random forest model" was retracted in 2025. Reasons: concerns about the results or conclusions; concerns about the peer review; concerns about the authorship.

Ren et al. (2022) [32] proposed two novel approaches to evaluate the predictability of carbon futures returns based on a wide range of factors. By employing dimensionality reduction techniques in their models, they identified the most influential predictive factors while considering potential variations in statistical significance across different carbon return quantiles. The findings underscore the importance of identifying appropriate carbon return predictive factors and understanding their impact, considering the carbon market’s dynamic nature. Li et al. (2022) [33] examined the impact of economic policy uncertainty on carbon emission allowance prices in the Chinese carbon emission trading market using non-linear models and asymmetric causality tests. The empirical results revealed that trade policy uncertainty and monetary policy uncertainty positively influence carbon emission allowance prices, whereas exchange rate policy uncertainty has a negative effect. Zhang et al. (2022) [34] conducted a comprehensive bibliometric analysis of the carbon neutrality theme, providing quantitative and visual insights into research progress and the evolution of research hotspots. The analysis highlighted the significance of low-carbon development as a prerequisite for achieving carbon neutrality, with an emphasis on emission reduction and carbon sinks.

In the realm of energy consumption, economic development, and carbon trading markets, Zhang et al. (2020) [35] undertook an assessment of the emissions trading scheme (ETS) to gauge its effectiveness and efficiency in curtailing carbon emissions. They also aimed to ascertain whether its implementation yielded concurrent benefits for both the economy and the environment. Their methodology involved the utilization of a differences-in-differences approach to evaluate the influence of ETS on carbon emissions and economic growth while scrutinizing its potential synergistic effects on these two aspects. In a separate study conducted by Zhang et al. (2022) [36], they devised an energy consumption permit allocation scheme grounded in principles of coordination, efficiency, and fairness. This scheme leveraged game theory alongside fixed cost allocation models and leader-follower game models. The study delved into the intricate dynamics between two interrelated market instruments within China’s Fujian province: the carbon emissions trading system and the energy consumption permit trading scheme. Kirikkaleli et al. (2022) [37] employed methodologies encompassing autoregressive distributed lag boundaries in a distinct investigation. Their primary objective was to explore the influence of financial development and renewable energy consumption on consumption-based carbon dioxide emissions in Chile. This analysis took into account factors such as economic growth and electricity consumption, offering a comprehensive perspective on the subject. Moving to a different aspect of research, Muhammad and Khan (2019) [38] conducted a multifaceted inquiry that examined the role played by factors including bilateral foreign direct investment, energy utilization, carbon dioxide emissions, and capital in the economic growth of Asian countries.

The article "Analysis of China’s carbon market price fluctuation and international carbon credit financing mechanism using random forest model" was retracted in 2025. Reasons: concerns about the results or conclusions; concerns about the peer review; concerns about the authorship.

Further details of these noteworthy studies are presented in Table 1.

**Table 1:** Research details on energy consumption, economic development, and carbon trading markets.

Author	Background	Methods	Findings	Summary
Zhang et al. (2020)	China introduced carbon ETS in seven pilot regions since 2013 to reduce industrial carbon emissions and address climate change.	Employed the differences-in-differences approach to assess the effectiveness of the ETS, analyzed industrial carbon emission data, and used data envelopment analysis to evaluate the operational efficiency of the seven ETS markets.	The implementation of the carbon emissions trading system significantly increased economic returns (13.6%) and reduced industrial CO_2_ emissions (24.2%). The average operational efficiency of the seven carbon emissions trading systems improved annually.	China’s carbon ETSs have significantly promoted economic growth and reduced emissions.
Zhang et al. (2022)	The Fujian province of China implemented both a carbon emissions trading system and an energy consumption permit trading scheme, and the interaction between these two market instruments could pose challenges.	Designed an energy consumption permit allocation scheme based on coordination, efficiency, and fairness principles using game theory and compared allocation structures between different cities and regional economic inequalities.	Under the consideration of optimal cross-efficiency, the allocation of energy consumption permits, and carbon emission permits is primarily dominated by economically prosperous coastal cities, which may exacerbate economic inequality between cities. However, when fairness principles are introduced, the allocation structure of energy consumption permits changes significantly, especially in underdeveloped cities. Mechanisms coordinating the carbon emissions trading system and energy consumption permit trading scheme can mitigate economic development inequality between cities.	Prioritizing the efficiency of energy consumption permit allocation over carbon emission permits is advantageous for energy conservation and emissions reduction.
Kirikkaleli, Güngör and Adebayo (2022)	The study focuses on consumption-based carbon dioxide emissions in Chile and explores the impact of financial development and renewable energy consumption while considering economic growth and electricity consumption.	Employed various analytical methods, including autoregressive distributed lag boundaries, fully modified ordinary least squares, dynamic ordinary least squares, and progressively transforming causal relationship tests, to assess the impact of various factors on carbon emissions.	Financial development and renewable energy consumption can reduce consumption-based carbon dioxide emissions, while economic growth and electricity consumption increase carbon emissions. The progressively transforming causal relationship test results are consistent with other estimation methods.	It is recommended that Chilean policymakers focus on the development of renewable energy and low-carbon technologies while limiting non-renewable energy consumption.
Muhammad and Khan (2019)	Emerging and developing economies increasingly attract foreign direct investment, while energy consumption, carbon emissions, and capital influence economic growth.	Utilized generalized method of moments, ordinary least squares regression, fixed effects, and random effects estimators, using cross-national data from 34 Asian host countries and 115 source countries between 2001 and 2012.	Energy consumption, inflow and outflow of foreign direct investment, carbon emissions, and capital play significant roles in the economic growth of Asian countries.	It is suggested that Asian countries improve energy utilization policies, encourage foreign investors to invest in Asian countries, and promote economic growth in the region.

The aforementioned studies aimed to explore the complex relationships among energy consumption, CO_2_ emissions, foreign direct investment, economic growth, and the impact of carbon emissions trading systems on carbon emissions and economic growth. They employed various methods, including the differences-in-differences approach, game theory models, autoregressive distributed lag boundaries, and generalized method of moments, to assess the influence of these factors on the economies and environments of different countries. In general, these studies found that financial development, renewable energy consumption, and foreign direct investment positively affect reducing carbon emissions and promoting economic growth. However, they also highlighted some challenges and inequalities. Substantial progress has been made in analyzing the volatility of carbon prices in the carbon trading market and the carbon credit financial market. The current market situation is characterized by an oversupply of freely allocated carbon emission allowances, resulting in reduced demand for additional carbon emission rights among companies to fulfill operational requirements. Consequently, pilot carbon trading markets exhibit low transaction volumes. As the carbon trading market is still in its early stages, data availability and quality may impose certain limitations, potentially impacting research on carbon price fluctuations and the carbon credit financial market, and leading to analytical constraints. Furthermore, limited research available on the intersection of carbon trading and international carbon credit financing, as well as the analysis of specific influencing factors in conjunction with case studies. To address these research gaps, this study aims to predict carbon price fluctuations, assisting companies and investors in formulating more informed investment strategies and mitigating risks.

The article "Analysis of China’s carbon market price fluctuation and international carbon credit financing mechanism using random forest model" was retracted in 2025. Reasons: concerns about the results or conclusions; concerns about the peer review; concerns about the authorship.

## 3 Research methodology

### 3.1 International carbon credit financing mechanism

Carbon credits form an integral part of the broader concept of green finance, which seeks to drive the transition to a more sustainable economy at the national and global levels, while also promoting ecological well-being. Green finance encompasses a range of economic activities facilitated by financial institutions, spanning areas such as energy conservation, environmental protection, clean energy, and green buildings. These activities include project operation, financial risk management, and project investment/financing. International carbon credit, as an extension of the original green credit system and model, is primarily structured around two low-carbon credit systems. The first system involves extending loans to low-carbon enterprises or supporting low-carbon projects through preferential loan interest rates. The second system entails granting loans to Certified Emission Reductions under the Clean Development Mechanism project through the platform of the global carbon rights trading market.

The article "Analysis of China’s carbon market price fluctuation and international carbon credit financing mechanism using random forest model" was retracted in 2025. Reasons: concerns about the results or conclusions; concerns about the peer review; concerns about the authorship.

Currently, Chinese commercial banks predominantly embrace the first variant of carbon credit, wherein they extend credit assistance to green and low-carbon enterprises. Carbon finance encompasses the business of pledging carbon emission rights as collateral for Renminbi (RMB) credit, which commercial banks offer to fulfill national policy requirements, green credit policy mandates, and regulatory authorities’ social responsibilities. This type of financing serves enterprises in their pursuits of emission reduction project implementation, technological transformation, upgrading, operational undertakings, and maintenance activities, among other objectives. This mode of financing is often accessed by entities possessing valid carbon emission quotas in the form of carbon emission units by carbon asset management companies responsible for administering and safeguarding carbon emission rights on behalf of third parties. Such candidates typically maintain basic or general deposit accounts with Chinese commercial banks.

The international carbon market has consistently led the way in pioneering innovative trading instruments for the carbon market. Carbon financial derivatives were among the pioneering additions to the EU’s carbon emissions trading system, propelling it to its current status as the world’s most extensive and representative carbon financial market. The augmentation of the carbon financial product portfolio has significantly fortified the carbon trading market’s capacity to function as a catalyst for key roles, such as price discovery, risk avoidance, and hedging. These functions, in turn, bolster the liquidity and market orientation of the carbon market while simultaneously promoting a more transparent carbon trading mechanism. Fig 1 depicts the fundamental theoretical mechanism of the carbon trading market.

**Fig 1:** Primary theoretical mechanism of the carbon trading market.

### 3.2 Carbon trading price forecast based on time series models

The objective of constructing carbon finance is to mitigate greenhouse gas emissions, such as carbon dioxide. However, before evaluating the effectiveness of carbon emission trading systems in curbing carbon dioxide emissions, it is imperative to conduct a comprehensive analysis of their emission reduction mechanisms. Carbon emissions trading encompasses five pivotal elements: total target, quota management, initial allocation, transaction price, and transaction subject. The synergistic interaction of these elements culminates in the achievement of emission reduction objectives facilitated by trading incentives, production curtailment, and the advancement of innovative green technologies. This study presents a corresponding schematic diagram, as illustrated in Fig 2, to provide a visual representation of the carbon emission trading process and its emission reduction mechanisms.

The article "Analysis of China’s carbon market price fluctuation and international carbon credit financing mechanism using random forest model" was retracted in 2025. Reasons: concerns about the results or conclusions; concerns about the peer review; concerns about the authorship.

**Fig 2:** Carbon emissions trading process and emission reduction mechanism.

Given that the data representing the carbon trading price series is organized as a time series, with each value corresponding to a specific time point, the sequencing of these values assumes paramount significance in data processing. It is imperative to recognize that a random partitioning of the dataset into distinct training and test sets is not unsuitable due to the inherent time-based structure of the data. Consequently, the approach employed in this study entails the utilization of a sequential temporal data point as the demarcation criterion. This procedure culminates in the division of the complete dataset into two distinct components: the designated training set and the test set. Specifically, the temporal extent allocated to the training set spans from August 1, 2015 to January 5, 2021. In parallel, the temporal coverage assigned to the test set covers the timeframe from January 6, 2021 to August 31, 2022. The pertinent market transaction price data pertaining to carbon emission rights is meticulously sourced from the Guotaian China Economic and Financial Research Database. The rate of return associated with the carbon transaction price is calculated by Eq (1).


$${Pr}_{t}\in ln\frac{P_{t}}{P_{t-1}}$$ (1)

In Eq (1), *Pr*_*t*_, *P*_*t*_, and *P*_*t*−1_ represent the current trading day’s price yield, the average transaction price, and the average price of the previous trading day, respectively.

Given the pronounced volatility and concentration manifesting within the realm of carbon emission allowance market trading price returns, marked by recurrent and substantial oscillations, the employment of the Autoregressive Integrated Moving Average (ARIMA) model emerges as particularly pertinent. This model possesses the capability to discern and encapsulate underlying trends and cyclic patterns intrinsic to time series data. Additionally, the Generalized Autoregressive Conditional Heteroskedasticity (GARCH) model emerges as a fitting choice due to its adeptness in accommodating the heteroskedastic nature of volatility. The harmonious fusion of these two models yields a holistic framework amenable to a more comprehensive and nuanced examination of alterations in carbon market price dynamics. It warrants emphasis that the use of both GARCH and ARIMA-type models enjoys a well-entrenched status within the financial field, substantiated by rigorous validation and extensive empirical scrutiny.

The article "Analysis of China’s carbon market price fluctuation and international carbon credit financing mechanism using random forest model" was retracted in 2025. Reasons: concerns about the results or conclusions; concerns about the peer review; concerns about the authorship.

In the context of time series data analysis, the imperative of establishing data stationarity assumes paramount significance. The presence of non-stationary time series data undermines the efficacy of regression models in their capacity to expound upon real-world phenomena. Consequently, a meticulous evaluation of the stationarity pertaining to trading price returns within the ambit of the nationwide unified carbon market is undertaken. This evaluation is carried out through the unit root Augmented Dickey-Fuller (ADF) test, as delineated in Table 2.

**Table 2:** Unit root test.

Category	ADF value	Confidence			P value	Conclusion
		1%	5%	10%		
National Unified Carbon Market	-11.2233	-3.5433	-2.8765	-2.3422	0.0001	smooth

The outcomes derived from the ADF unit root test unveil a state of stability within the yield of the transaction price in the unified carbon trading market. This state of stability, substantiated by the null hypothesis rejection at a 99% confidence threshold, lends credence to the robustness of the examined data. Subsequent to this evaluation, the derivation of residuals through the mean equation. The results of the heteroscedasticity test conducted on these residuals are presented in Table 3.

**Table 3:** GARCH heteroscedasticity test for volatility.

Category	F-statistic	Probability value (P)	T * R^2^ statistic	Probability value (P)
National Unified Carbon Market	8.8344	0.0005	14.3222	0.0005

Table 3 conspicuously demonstrates that the established mean equation exhibits a noticeable presence of heteroscedasticity, thereby fulfilling the prerequisite for employing the GARCH model to examine the volatility of carbon trading prices and returns. Thus, the utilization of GARCH and ARIMA models to investigate the price volatility in the unified carbon market is justifiable and appropriate.

A typical standardized GARCH(1,1) model is formulated as:

$$y_{t}=x^{T}\gamma +u_{t}$$ (2)

$$u_{t}=\sigma_{t}\varepsilon_{t}$$ (3)

$$\sigma_{t}^{2}=\beta_{0}+\beta_{1}u_{\left(t-1\right)}^{2}+\beta_{2}\sigma_{\left(t-1\right)}^{2}$$ (4)

Eq (2) delineates the mean value equation integral to the GARCH(1,1) model, wherein *x* represents the explanatory variable, *γ* signifies the coefficient of the variable, *u*_*t*_ denotes the residual term, and *ε*_*t*_ represents a disturbance term that follows a specific distribution, such as normal distribution and t-distribution. Eq (4) illustrates the conditional heteroscedasticity equation in the GARCH(1,1) model, which characterizes the fluctuation trend of the residual term *u*_*t*_. In Eq (4), *β*_*1*_ and *β*_*2*_ denote the coefficients that measure the strength and duration of the impacts on the conditional variance. Notably, augmented values of these coefficients indicate heightened magnitudes of impacts and extended durations.

The article "Analysis of China’s carbon market price fluctuation and international carbon credit financing mechanism using random forest model" was retracted in 2025. Reasons: concerns about the results or conclusions; concerns about the peer review; concerns about the authorship.

Ensuring the stationarity of the data is a pivotal step in upholding the reliability of sequence modeling. Although a cursory examination of the time series plot can provide some insights into the stability of carbon trading trends, it is a subjective approach. Hence, the ADF test, recognized for its unit root test assessment capability, is employed to evaluate the stationarity of the carbon price series. The significance level for this assessment is set at 0.05, imparting statistical rigor to the evaluation. The ADF test augments the original Dickey-Fuller test by extending its applicability beyond first-order scenarios. It accommodates high-order lagged correlations in the series. The primary purpose is to discern the presence of a unit root in the sequence. Specifically, the identification of sequence stability indicates the absence of a unit root, signifying stationarity. Conversely, the detection of a unit root suggests non-stationarity. Following the transformation of the non-stationary time series into a stationary form via differencing, the groundwork is laid for the construction of an ARIMA model. This model facilitates the revelation of underlying patterns inherent in the series.

In ARIMA models, a prevailing assumption resides in the constancy of the variance of the disturbance term. However, circumstances often arise where the variance of this term, especially concerning temporal fluctuations, deviates from a state of constancy. This underscores the imperative of factoring in the volatility characteristic when studying time series models. Relying solely on autocorrelation and partial autocorrelation diagrams to discern the optimal model order can be intricate. Therefore, this study opts to instantiate an ARIMA(1,1,1) model. Moreover, using a general GARCH model with a high order can potentially undermine model precision and introduce heightened instability. In contrast, the GARCH(1,1) model has gained recognition for its enhanced stability. Hence, this study chooses to combine the ARIMA(1,1,1) model with the GARCH(1,1) model to formulate an integrated ARIMA(1,1,1)-GARCH(1,1) model for predicting carbon trading prices. This model can be expressed as:

$$\left\{\begin{array}{ll} y_{t}=0.84y_{t-1}+0.16y_{t-2}+\varepsilon_{t}+\varepsilon_{t-1} & \left(5\right)\\ \varepsilon_{t}=0.18\varepsilon_{t-1}+v_{t} & \left(6\right)\\ v_{t}=\sqrt{h_{t}}e_{t} & \left(7\right)\\ h_{t}=0.85h_{t-1}+0.11v_{t-1}^{2} & \left(8\right) \end{array}\right.$$

The ARIMA(1,1,1)-GARCH(1,1) model finds its frequent application within univariate time series analysis. However, the intricacies of real-world scenarios frequently entail the influence of multiple sequences upon the evolution of a given sequence. Consequently, the exigency arises for the adoption of techniques within the realm of multivariate time series analysis. An established solution in this context is the ARIMAX model. It encompasses multiple time series variables to capture the dynamic regression effects. Fig 3 reveals the steps involved in formulating the ARIMAX model.

The article "Analysis of China’s carbon market price fluctuation and international carbon credit financing mechanism using random forest model" was retracted in 2025. Reasons: concerns about the results or conclusions; concerns about the peer review; concerns about the authorship.

**Fig 3:** ARIMAX model modeling flow chart.

Fig 3 delineates a systematic progression encompassing pivotal steps within the ARIMAX modeling framework. These steps include the following steps:

1. Stationarity assessment and transformation: Commencing with the scrutiny of multiple original sequences, the initial focus resides on subjecting them to stationarity tests. Should these sequences demonstrate non-stationary, essential transformations are employed to render them stationary, thus ensuring robust analysis.
2. Individual ARMA Modeling: The subsequent phase entails the distinct modeling of the ARMA model for each stationary input variable sequence {*x*_*it*−1_} and response sequence {*y*_*t*_}. This process engenders the derivation of their respective residual sequences {*ε*_*it*_} and {$\varepsilon_{y_{it}}$};
3. Cross-correlation coefficient evaluation: A comprehensive cross-correlation coefficient evaluation is then conducted on the residual sequence {*ε*_*t*_}, interfacing it with the meticulous construction of the ARIMAX model.
4. White noise assessment: The final step encompasses a meticulous white noise assessment of the residual sequence {*ε*_*t*_}. Conformance with established criteria for a white noise sequence renders it deemed satisfactory. In instances where compliance is not met, recalibration of parameters is undertaken to rectify the disparity.

### 3.3 Analysis of influencing factors of carbon market price fluctuation based on random forest algorithm

This study combines the random forest algorithm and the quantile regression method to comprehensively analyze the factors influencing price fluctuations in the carbon market. While the time series model is utilized to predict the price fluctuations in the carbon trading market, it remains imperative to acknowledge the intricate interplay of diverse factors contributing to these dynamic fluctuations. Accordingly, this section focuses on investigating the underlying determinants shaping price oscillations in the carbon market. This endeavor is enabled by the judicious application of both the random forest algorithm and quantile regression method, furnishing a holistic analytical approach. Upon conducting research, it has been determined that fluctuations in carbon market prices pose a consequential risk that can dampen the enthusiasm of enterprises, units, and other participants. This potential dampening effect underscores the significance of effective carbon emission reduction efforts. This study investigates the utilization of data mining methods for identifying influential factors affecting carbon market prices. The overarching objective is the establishment of regulation mechanisms fostering stability in market prices, thereby promoting the development of the carbon trading market in the era of big data. The research object of this study comprises valid carbon trading data records from August 1, 2015, to August 31, 2022, each captured at a daily frequency. Non-trading days, such as holidays, have been prudently excluded from consideration, yielding a corpus of 1235 meticulously curated data entries. These data emanate from authoritative sources, including the Guotaian database, the Ruisi database, and the China Statistical Yearbook. This study focuses on four robustly active markets, namely Beijing, Guangdong, Shenzhen, and Hubei, encompassing abundant data samples. This focused market scope facilitates the rigors of feature screening to ensure research validity. Table 4 presents some data indicators used in the analysis. This study focuses on historical data from the carbon pilot market to select relevant features. These selected features are then used to forecast the price data of the nationwide unified carbon market. The accuracy of the predictions is evaluated by comparing them with actual values, thereby assessing the suitability of the selected features for predicting carbon emission trading prices in the nationwide unified carbon market. The research scope encompasses China’s carbon market price fluctuations and the international carbon credit financing mechanism, spanning from August 1, 2015, to August 31, 2022.

The article "Analysis of China’s carbon market price fluctuation and international carbon credit financing mechanism using random forest model" was retracted in 2025. Reasons: concerns about the results or conclusions; concerns about the peer review; concerns about the authorship.

**Table 4:** Selection and description of main data indicators.

Category	Specific indicators	Indicator number
Traditional energy	Ex-factory price index of oil and natural gas industry	X1
	Daqing Crude Oil Price Index	X2
	Foreign WTI crude oil futures price	X3
	Spot price of Brent crude oil	X4
New energy	China Coastal Coal Freight Index	X5
	Proportion of national hydropower generation	X6
	Proportion of nuclear power generation in the country	X7
Natural environment	Air quality index	X8
	average temperature	X9
Carbon financial market	carbon yield	X10
	Growth rate of carbon trading volume	X11
	Natural Gas Futures Closing Price	X12
Industry index	Shanghai Industrial Index	X13
	Shanghai Stock Exchange Energy Index	X14
	SSE Industrials Index	X15
	Shenzhen Industrial Index	X16
	CSI Energy Index	X17
Macro environment	Chinese government bond yield table	X18
	Foreign currency to RMB central parity	X19
	S&P 500 Index	X20

With the ever-evolving advancements in big data technology, machine learning algorithms have garnered escalating prominence in the realm of economic and social research. This phenomenon holds particularly true within the intricate domain of carbon trading pricing. The multifaceted nature of carbon trading pricing issues embodies intricate interactions between society and nature. This intricate nexus is influenced by numerous factors simultaneously. However, concomitant with the proliferation of these factors, the analysis of data may encounter the challenge of the curse of dimensionality. To surmount this issue, this study incorporates the deployment of the random forest model. This model emerges as a potent tool uniquely positioned to effectively circumvent the complexities posed by the curse of dimensionality. By leveraging the tenets of factor feature importance, the random forest model facilitates the identification of critical factors among the many influencing factors. Moreover, the machine learning model conducts information mining based on sample data. This model operates within the realm of continuous learning and iterative refinement, culminating in the identification and elucidation of optimal strategies.

Bagging decision trees, exemplified by the widely utilized random forests, represent a technique for estimating the importance of features. This valuation offers a foundation upon which to undertake feature selection endeavors by eliminating attributes exhibiting low scores while retaining those with high scores. This approach essentially encompasses an algorithm combining Bagging theory and Random Subspace principles. Fig 4 visually represents the specific algorithm flow for random forests.

**Fig 4:** Random forest decision flow.

As illustrated in Fig 4, the random forest algorithm unfolds through a series of well-defined steps:

1. Replacement sampling for diverse training sets: The algorithm initiates by subjecting the prevailing training sample data to a regimen of replacement sampling. This process engenders the creation of multiple sample sets, each encompassing n samples drawn in each iteration.
2. Candidate feature selection via random sampling: Within this stage, m candidate features are selectively drawn from the feature pool under consideration. Subsequently, these features are subjected to rigorous training sample analysis, facilitating the identification of optimal features through feature selection.
3. Construction of multiple decision trees: This phase involves the deployment of each sample set to train a dedicated decision tree. The cumulative outcome is the emergence of an ensemble of multiple decision trees.
4. Voting mechanism for final decision output: Upon the creation of a certain number of decision trees, the algorithm embarks upon a deliberative voting process. This entails the amalgamation of the final decision result of the random forest selected based on the outcome with the highest number of votes.

The article "Analysis of China’s carbon market price fluctuation and international carbon credit financing mechanism using random forest model" was retracted in 2025. Reasons: concerns about the results or conclusions; concerns about the peer review; concerns about the authorship.

Eq (9) indicates the convergence of the random forest generalization error GE* for all random variable sequences *θ*_1_, *θ*_2_, …, *θ*_*k*_ as the number *N* in the decision tree *k*(*x*_1_), *k*(*x*_2_), …, *k*(*x*_*n*_) increases.


$$\underset{N\to \infty }{lim}GE^{*}=P_{xy}\{P_{\theta }[k(x,\theta )=Y]-\underset{j\neq Y}{max}P_{\theta }(k(x,\theta )=j)<0\}$$ (9)

In Eq (9), *y* represents the correct classification vector; *j* stands for the vector that has not been classified correctly; *P*_*xy*_ signifies the joint probability of random variables *x* and *y*; *P*_*θ*_ denotes the probability of random variables.*θ*

In a random forest framework, each decision tree comprises multiple decision nodes. An appraisal of its significance becomes imperative to discern the influence wielded by a particular feature within each decision tree. This contribution is ascertained by quantifying the difference in the Gini index (Gini) before and after the branching of the feature at a particular node. Analogous calculations are extensible to ascertain the contribution of other features. Subsequently, the normalized contribution of a feature can be obtained by dividing the alteration in the Gini index of that feature by the sum of the changes witnessed across all features. Hence, the importance of each node *i* can be calculated using Eq (10).


$$m_{i}=\mu_{i}∙G_{i}-\mu_{ileft}∙G_{ileft}-\mu_{iright}∙G_{iright}\}$$ (10)

In Eq (10), *μ*_*i*_, *μ*_*ileft*_, and *μ*_*iright*_ denote the proportions of training samples of node *i* and its left and right nodes, respectively, with respect to the total sample size, representing the Gini coefficients of node *i* and its left and right nodes. Eq (11) calculates the importance of a certain feature.


$$f_{i}=\frac{\sum_{j\in nodes\;split\;on\;feature\;i}m_{j}}{\sum_{k\in all\;nodes}m_{k}}$$ (11)

However, the features garnered through the comprehensive screening methods might exhibit a notable degree of correlation, potentially instigating overfitting in subsequent modeling. Therefore, a crucial step entails subjecting these variables to an independence test. This process facilitates the retention of the variable that yields the highest contribution among a pair of closely associated variables while concurrently discarding the secondary variable. Here, the top 10 variables are selected as the screening results of the second-stage screening process. Next, a prediction model is built based on the random forest algorithm, and the root mean square error (RMSE), mean square error (MSE), mean absolute error (MAE), and goodness of fit (R) are used as evaluation indicators:

$$MSE=\frac{1}{n}\sum_{t=1}^{n}{\left(y_{t}-y_{t}^{*}\right)}^{2}$$ (12)

$$RMSE=\sqrt{\frac{1}{n}\sum_{t=1}^{n}{\left(y_{t}-y_{t}^{*}\right)}^{2}}$$ (13)

$$MAE=\frac{1}{n}\sum_{t=1}^{n}\left|y_{t}-y_{t}^{*}\right|$$ (14)

$$R^{2}=1-\frac{MSE(y_{t},y_{t}^{*})}{Var(y_{t})}$$ (15)

where *y*_*t*_ represents the actual value, and $y_{t}^{*}$ signifies the predicted value.

The article "Analysis of China’s carbon market price fluctuation and international carbon credit financing mechanism using random forest model" was retracted in 2025. Reasons: concerns about the results or conclusions; concerns about the peer review; concerns about the authorship.

The intricate interplay of myriad factors impact the price of the carbon market, and their influence on carbon trading prices may exhibit a non-linear relationship, deviating from strict linearity. As a result, this study employs a quantile regression model to investigate the distinct effects of the key factors that have been identified through screening at various quantile points on the price of carbon trading, as illustrated in Eq (16).


$$y_{i}=x_{i}\beta (\theta )+\epsilon (\theta )$$ (16)

In Eq (16), *y*_*i*_ and *x*_*i*_ represent the explained variable and explanatory variable; *θ* refers to the quantile point; *ϵ*(*θ*) denotes the random disturbance item; *β*(*θ*) indicates the estimated coefficient under the quantile point *θ*, which is calculated according to:

$$\beta (\theta )=\underset{\beta }{min\;}\sum_{i}\rho_{\theta }(y_{i}-x\beta (\theta )),\theta \in (0,1)$$ (17)

Eq (18) describes *ρ*_*θ*_ in Eq (17).


ρθ={μθ,μ⩾0μ(θ-1),μ<0 (18)

Meanwhile, for given variables *y*_*i*_ and *x*_*i*_, the quantile function *θ* is expressed as Eq (19).


$$y_{\theta }(x_{i})=x_{i}\beta (\theta )$$ (19)

## 4 Results and discussion

### 4.1 Performance comparison of different time series forecasting models

Given the idiosyncratic attributes of the carbon emission rights market, marked by peak values and heavy-tailed distributions in transaction prices, this study incorporates the construction of a GARCH model under various distribution conditions, including the normal distribution, for testing purposes. The corresponding results are presented in Table 5.

**Table 5:** Test analysis based on the GARCH family model.

Model	Distribution	*ω*	A	β	DOF /GED
GARCH	Normal distribution	0.002047*** (0.000309) (0.0000)	0.791542 ** (0.371513) (0.0331)	-2.07409** (0.093680) (0.0268)	/
	T-distribution	0.002360 (0.004658) (0.6124)	1.948148 (4.044858) (0.6301)	0.068700 (0.173989) (0.6927)	2.252968
	GED distribution	0.001166** (0.000592) (0.0487)	0.605696 (0.775743) (0.4349)	0.167443 (0.335228) (0.6174)	0.646590

Table 5 indicates that all parameters in the model for the national unified carbon market are statistically significant at the 95% confidence interval. Concurrently, these parameters substantively satisfy the condition of α + β < 1. This outcome implies that the unified carbon market distinctly embodies the hallmarks of peak values and heavy-tailed distributions. This characterization sheds light on the dynamic landscape of price fluctuations, further unveiling a discernible undercurrent of persistence. Furthermore, a heteroscedasticity test is conducted on the GARCH model under a normal distribution, yielding non-significant results. This profound observation underscores the competence of the model adequately captures the ARCH effect of the carbon emission rights market’s transaction price return sequence under this distribution.

The article "Analysis of China’s carbon market price fluctuation and international carbon credit financing mechanism using random forest model" was retracted in 2025. Reasons: concerns about the results or conclusions; concerns about the peer review; concerns about the authorship.

Python is employed to visually represent the carbon trading price series from 2015 to 2022 and its first-order difference sequence, as depicted in Fig 5.

**Fig 5:** Timing diagram of carbon trading price (a. original sequence; b. first-order difference sequence).

The visualization presented in Fig 5 distinctly portrays the marked volatility characterizing the carbon market’s transaction price. Fig 6 presents a comparison to further assess the prediction performance of different time series models discussed earlier.

**Fig 6:** Comparison of real value and predicted value.

Fig 6 highlights the discrepancy between the predicted time series trajectory generated by the prediction model and the actual result. Notably, a distinctive refinement surface upon subjecting the dataset to the rigors of the Least absolute shrinkage and selection operator (LASSO) filtering. In this context, the ARIMAX model outperforms the ARIMA(1,1,1)-GARCH(1,1) model in terms of predictive efficacy and prediction error. The ARIMA(1,1,1)-GARCH(1,1) model registers a relatively lower R^2^ value of 0.68 and concurrently exhibits notable accuracy with an R^2^ value of 0.85. The ARIMAX(LASSO) model also yields favorable results for MSE, RMSE, and MAE, quantified at 0.022, 0.1344, and 0.1543, respectively. These values are significantly close to the ideal of zero, thereby underscoring the superior performance of the ARIMAX(LASSO) model compared to its contemporaries.

### 4.2 Prediction of carbon market price based on random forest

The transaction price of carbon emission rights in the national unified carbon market is forecasted using a random forest prediction model created using the screening features. Fig 7 displays the visual outcomes.

The article "Analysis of China’s carbon market price fluctuation and international carbon credit financing mechanism using random forest model" was retracted in 2025. Reasons: concerns about the results or conclusions; concerns about the peer review; concerns about the authorship.

**Fig 7:** Prediction and evaluation results of random forest model.

Fig 7 displays the national carbon market price prediction model built using the selected features boasting a goodness of fit of 0.9567. The data indicates that the features’ robust explanatory capacity for the transaction price of the carbon emission rights market affirming the model’s data comprehension. The resulting impact is satisfactory. Meanwhile, with MSE, RMSE, and MAE at 0.032, 0.1874, and 0.1324, correspondingly, the model demonstrates close alignment between actual outcomes, underscoring its sound prediction accuracy. Fig 8 depicts the random forest model’s regression procedure.

**Fig 8:** Visual regression process of random forest.

Empirical insights into the identical factor, underpinning different quantile regression analyses, are gleaned through the formulation of ten distinct quantile regression models spanning quantiles from 0.05 to 0.95. This discerning analytical approach culminates in the elucidation of these findings, visually encapsulated in Figs 9 and 10.

**Fig 9:** Empirical results under different quantiles (q = 0.05~0.45).

**Fig 10:** Empirical results under different quantiles (q = 0.55~0.95).

Figs 9 and 10 showcase abscissae labeled as “R1R10,” delineating the discernible factors wielding impact. This compilation encompasses the Shenzhen Stock Exchange Industrial Index, the Manufacturing Purchasing Managers Index, the Margin and Securities Lending Balance, the Futures Closing Price (Steam Coal), the Oil Industrial Products Exit Price index, the ex-factory price index of coal and coking industrial products, the SSE 50, foreign currency-to-RMB exchange rate, turnover growth rate, and the latest closing price of natural gas futures (New York). Figs 9 and 10 underscore the pivotal role assumed by a constellation of factors. Specifically, the CSI 300 Industrial Index, the Purchasing Managers’ Index for Manufacturing, the Futures Closing Price for Thermal Coal, the Producer Price Index for Coal and Coke Industries, and the Exchange Rate of Foreign Currency versus the RMB all have significant impacts on trading prices in the carbon market at the 0.01% confidence level. These pronounced impacts substantiate the pivotal standing of these elements in the carbon market. Moreover, the empirical terrain delineates the influence of the Producer Price Index for Coal and Coke Industries and the Producer Price Index for Petroleum and Coal Products, both exercising a negative influence on carbon trading prices. Notably, the heightened rate of trade volume yields comparatively nuanced effects, attaining statistical significance solely at the 0.05, 0.15, and 0.35 quantile points, thus manifesting a less conspicuous imprint within this intricate ecosystem.

The article "Analysis of China’s carbon market price fluctuation and international carbon credit financing mechanism using random forest model" was retracted in 2025. Reasons: concerns about the results or conclusions; concerns about the peer review; concerns about the authorship.

Similarly, several macroeconomic indicators, including the Shenzhen Industrial Industry Index, the Manufacturing Purchasing Managers’ Index, the Producer Price Index of Petroleum Industrial Products, and the Producer Price Index of Coal and Coke Industrial Products, manifest a notable negative correlation with the dependent variable. The correlation’s robust statistical significance further supports their impact on the model. Moreover, variables such as margin trading and short selling balance, foreign exchange rates against the Chinese RMB, and the recent closing price of natural gas futures (New York) evince differential effects on the dependent variable based on different quantiles. The Shanghai 50 Index consistently projects a positive influence on the dependent variable, maintaining its statistical significance across all quantiles. In contrast, the impact of the growth rate of trading volume assumes a conspicuously mutable disposition, displaying substantial variation across disparate quantiles and lacking a consistent pattern of influence.

### 4.3 Discussion

The analysis of empirical data reveals that both carbon trading and stock market data are often influenced by multiple factors, and there may exist complex non-linear relationships among these factors. The supply and demand dynamics of carbon emissions quotas may exhibit diverse non-linear patterns at different price levels. Similarly, in the stock market, factors such as investor sentiment and market expectations can also have non-linear effects on stock prices. Non-linear models, such as random forests, are better equipped to capture this complexity, thereby enhancing their ability to fit the data. Moreover, both carbon trading and stock market data typically have high dimensions involving multiple influencing factors. Traditional linear models are susceptible to overfitting in such high-dimensional data, whereas the random forest model is more adept at generalizing on high-dimensional data, thus reducing the risk of overfitting.

The preceding investigation has discerned a multitude of factors that exert influence on price fluctuations in the carbon trading market. Therefore, when conducting carbon credit and carbon finance business, a holistic consideration of these influencing factors assumes paramount importance. This strategic approach ensures the preservation of equilibrium within carbon market prices. Pertinently, analogous inquiries have been undertaken by Zhou et al. (2022) [39]. They built numerous one-step-ahead predictors based on an empirical mode decomposition of adaptive noise and long-short-term memory recurrent neural networks. These endeavors were founded on the closing prices of the Guangzhou carbon emissions trading plan from 2014 to 2021. In a similar vein, Sun and Huang (2020) [40] proposed a novel hybrid model for carbon price forecasting. This innovative paradigm incorporated a quadratic decomposition algorithm while harnessing a genetic algorithm-optimized backpropagation neural network model for prediction. Their model outperformed other comparative models in empirical analyses rooted in the Hubei market. Furthermore, Razzaq et al. (2022) [41] employed cross-quantitative diagrams and rolling window causality methods to dissect the asymmetric dependence structure and directional predictability of China’s carbon trading market. This examination was facilitated from the perspective of total volume and industry. These findings indicate the existence of various non-linear relationships in carbon trading and stock market data, underscoring the necessity of studying asymmetric behaviors to explore complex relationships, bolstering the pertinence and efficacy of this study.

The article "Analysis of China’s carbon market price fluctuation and international carbon credit financing mechanism using random forest model" was retracted in 2025. Reasons: concerns about the results or conclusions; concerns about the peer review; concerns about the authorship.

## 5 Conclusion

This study addresses the importance of adopting suitable methods and models to predict carbon market trading prices effectively, considering the volatility risks associated with carbon trading. It focuses on exploring the operation principles of the international carbon credit financing mechanism and applies time series models for price prediction. The research employs an ARIMA(1,1,1)-GARCH(1,1) joint model, integrating GARCH and ARIMA-type models alongside a multivariate dynamic regression ARIMAX model to analyze carbon market price volatility. A data indicator system is constructed, encompassing various influencing factors, and the random forest algorithm is utilized for feature selection, retaining high-score features and eliminating low-score features. Furthermore, quantile regression models are used to investigate the specific impact of key factors at different quantile levels on carbon trading prices. One of the research gaps addressed in this study pertains to the relationship between Chinese carbon market price fluctuations and the international carbon credit financing mechanism. By providing a novel approach to exploring this relationship, this research contributes to filling the research gap in related fields.

The theoretical contribution of this study primarily lies in the integration of time series modeling and machine learning for a deeper understanding of carbon market price fluctuations. The study makes a theoretical contribution by introducing an approach that integrates time series modeling and machine learning techniques. By combining the ARIMA(1,1,1)-GARCH(1,1) model with the random forest algorithm, this study innovatively addresses the prediction of carbon market price volatility. This approach holds promise for applications in forecasting other financial markets, providing new insights into time series analysis in various domains. This study gains a deeper understanding of the interrelationship between these two domains through the comprehensive analysis of multi-dimensional data, including data from two distinct domains: carbon market price fluctuations and international carbon credit financing mechanisms. This theoretical contribution provides a solid foundation for further research into the operation of carbon markets and international carbon credit financing mechanisms. The practical contributions of this study are of significant importance to practitioners in the carbon market and carbon credit financing fields. The proposed ARIMA(1,1,1)-GARCH(1,1) model demonstrates excellent performance in forecasting time series data. This advantage offers market participants a highly accurate tool for price prediction. Practitioners can leverage this model to plan their trading strategies better, reduce market risks, and enhance decision-making efficiency. This optimization holds practical value for carbon market investors, asset managers, and intermediaries. Given that carbon market price fluctuations can pose substantial financial risks, the high-accuracy price forecasting model presented in the study helps practitioners manage these risks effectively. Financial institutions and businesses can use this model to formulate risk mitigation strategies, mitigating the adverse impact of price fluctuations on their financial positions. As carbon markets evolve, policymakers need a better understanding of market operations and price trends to formulate effective policies and regulatory measures. The price forecasting model and data analysis methods presented in the study offer government agencies powerful decision support tools, aiding in the optimization of carbon market policy frameworks. The study provides practitioners with a more comprehensive market insight by synthesizing data on carbon market price fluctuations and international carbon credit financing mechanisms. This enhanced understanding helps investors better grasp the complexity of the carbon market, seize market opportunities, and reduce uncertainty. In summary, this study provides powerful tools and knowledge for practitioners in the carbon market and carbon credit financing fields, facilitating a better understanding of market dynamics, risk management, decision-making, and the advancement of the field. Ultimately, these contributions support the realization of a low-carbon economy and further progress in endeavors aimed at mitigating climate change.

The article "Analysis of China’s carbon market price fluctuation and international carbon credit financing mechanism using random forest model" was retracted in 2025. Reasons: concerns about the results or conclusions; concerns about the peer review; concerns about the authorship.

This study acknowledges certain limitations. The carbon market and carbon credit financing mechanisms are subject to dynamic changes over time, which can influence prices and mechanisms. The research’s time span might be considered relatively short, potentially limiting its ability to fully capture long-term trends and influencing factors. For future investigations, it is recommended to extend the data collection period, incorporating data from more years, particularly spanning multiple economic cycles. This approach would provide a comprehensive understanding of the variations and trends in carbon market prices and carbon credit financing mechanisms during different economic phases. Such extended research efforts will yield more robust and insightful findings for policymakers and stakeholders in the carbon market domain.

## Supporting information

S1 Data (XLSX)

## References

[1] Maestre-AndrésS, DrewsS, van den BerghJ. Perceived fairness and public acceptability of carbon pricing: a review of the literature[J]. Climate policy, 2019, 19(9): 1186–1204.

[2] JiaZ, LinB. Rethinking the choice of carbon tax and carbon trading in China[J]. Technological Forecasting and Social Change, 2020, 159: 120187.

[3] LinB, JiaZ. What are the main factors affecting carbon price in Emission Trading Scheme? A case study in China[J]. Science of the Total Environment, 2019, 654: 525–534. doi: 10.1016/j.scitotenv.2018.11.106 30447591

[4] GreenJ F. Does carbon pricing reduce emissions? A review of ex-post analyzes[J]. Environmental Research Letters, 2021, 16(4): 043004.

[5] XingE, ShiC, ZhangJ, et al. Double third-party recycling closed-loop supply chain decision under the perspective of carbon trading[J]. Journal of Cleaner Production, 2020, 259: 120651.

[6] WooJ, FatimaR, KibertCJ, et al. Applying blockchain technology for building energy performance measurement, reporting, and verification (MRV) and the carbon credit market: A review of the literature[J]. Building and Environment, 2021, 205: 108199.

[7] ZhuB, YeS, HanD, et al. A multiscale analysis for carbon price drivers[J]. Energy Economics, 2019, 78: 202–216.

[8] van der GaastW, SikkemaR, VohrerM. The contribution of forest carbon credit projects to addressing the climate change challenge[J]. Climate Policy, 2018, 18(1): 42–48.

[9] SkovgaardJ, FerrariSS, KnaggårdÅ. Mapping and clustering the adoption of carbon pricing policies: what policies price carbon and why? [J]. Climate Policy, 2019, 19(9): 1173–1185.

The article "Analysis of China’s carbon market price fluctuation and international carbon credit financing mechanism using random forest model" was retracted in 2025. Reasons: concerns about the results or conclusions; concerns about the peer review; concerns about the authorship.

[10] AnjosMF, FeijooF, SankaranarayananS. A multinational carbon-credit market integrating distinct national carbon allowance strategies[J]. Applied Energy, 2022, 319: 119181.

[11] LiuJ, WangP, ChenH, et al. A combination forecasting model based on hybrid interval multi-scale decomposition: Application to interval-valued carbon price forecasting[J]. Expert Systems with Applications, 2022, 191: 116267.

[12] TianC, HaoY. Point and interval forecasting for carbon price based on an improved analysis-forecast system[J]. Applied Mathematical Modeling, 2020, 79: 126–144.

[13] BlancS, AccastelloC, BianchiE, et al. An integrated approach to assess carbon credit from improved forest management[J]. Journal of Sustainable Forestry, 2019, 38(1): 31–45.

[14] WenF, ZhaoL, HeS, et al. Asymmetric relationship between carbon emission trading market and stock market: evidences from China[J]. Energy Economics, 2020, 91: 104850.

[15] DemiralayS, GencerHG, BayraciS. Carbon credit futures as an emerging asset: Hedging, diversification and downside risks[J]. Energy Economics, 2022, 113: 106196.

[16] FanX, ChenK, ChenY J. Is price commitment a better solution to control carbon emissions and promote technology investment?[J]. Management Science, 2023, 69(1): 325–341.

[17] TangBJ, JiCJ, HuYJ, et al. Optimal carbon allowance price in China’s carbon emission trading system: Perspective from the multi-sectoral marginal abatement cost[J]. Journal of Cleaner Production, 2020, 253: 119945.

[18] LyuJ, CaoM, WuK, et al. Price volatility in the carbon market in China[J]. Journal of Cleaner Production, 2020, 255: 120171.

[19] LvM, BaiM. Evaluation of China’s carbon emission trading policy from corporate innovation[J]. Finance Research Letters, 2021, 39: 101565.

[20] HuangY, DaiX, WangQ, et al. A hybrid model for carbon price forecasting using GARCH and long short-term memory network[J]. Applied Energy, 2021, 285: 116485.

[21] SongY, LiuT, LiangD, et al. A fuzzy stochastic model for carbon price prediction under the effect of demand-related policy in China’s carbon market[J]. Ecological Economics, 2019, 157: 253–265.

[22] LiL, YeF, LiY, et al. How will the Chinese Certified Emission Reduction scheme save cost for the national carbon trading system? [J]. Journal of environmental management, 2019, 244: 99–109. doi: 10.1016/j.jenvman.2019.04.100 31108316

[23] SiyalS, XinC, UmraniWA, et al. How do leaders influence innovation and creativity in employees? The mediating role of intrinsic motivation[J]. Administration & Society, 2021, 53(9): 1337–1361.

[24] HuM, ZhongY, XieS, et al. Fuzzy system based medical image processing for brain disease prediction[J]. Frontiers in Neuroscience, 2021, 15: 714318. doi: 10.3389/fnins.2021.714318 34393718 PMC8361453

The article "Analysis of China’s carbon market price fluctuation and international carbon credit financing mechanism using random forest model" was retracted in 2025. Reasons: concerns about the results or conclusions; concerns about the peer review; concerns about the authorship.

[25] DavoodiS, ThanhHV, WoodDA, et al. Machine-learning models to predict hydrogen uptake of porous carbon materials from influential variables[J]. Separation and Purification Technology, 2023, 316: 123807.

[26] LuH, MaX, HuangK, et al. Carbon trading volume and price forecasting in China using multiple machine learning models[J]. Journal of Cleaner Production, 2020, 249: 119386.

[27] HaoY, TianC, WuC. Modeling of carbon price in two real carbon trading markets[J]. Journal of Cleaner Production, 2020, 244: 118556.

[28] CaiW, YeP. Does carbon emission trading improve low-carbon technical efficiency? Evidence from China[J]. Sustainable Production and Consumption, 2022, 29: 46–56.

[29] VenmansF, EllisJ, NachtigallD. Carbon pricing and competitiveness: are they at odds? [J]. Climate Policy, 2020, 20(9): 1070–1091.

[30] HuangY, HeZ. Carbon price forecasting with optimization prediction method based on unstructured combination[J]. Science of the Total Environment, 2020, 725: 138350. doi: 10.1016/j.scitotenv.2020.138350 32304964

[31] NiuX, WangJ, ZhangL. Carbon price forecasting system based on error correction and divide-conquer strategies[J]. Applied Soft Computing, 2022, 118: 107935.

[32] RenX, DuanK, TaoL, et al. Carbon prices forecasting in quantiles[J]. Energy Economics, 2022, 108: 105862.

[33] LiX, LiZ, SuCW, et al. Exploring the asymmetric impact of economic policy uncertainty on China’s carbon emissions trading market price: Do different types of uncertainty matter?[J]. Technological Forecasting and Social Change, 2022, 178: 121601.

[34] ZhangZ, HuG, MuX, et al. From low carbon to carbon neutrality: A bibliometric analysis of the status, evolution and development trend[J]. Journal of Environmental Management, 2022, 322: 116087. doi: 10.1016/j.jenvman.2022.116087 36041302

[35] ZhangW, LiJ, LiG, et al. Emission reduction effect and carbon market efficiency of carbon emissions trading policy in China[J]. Energy, 2020, 196: 117117.

[36] ZhangY, WeiJ, GaoQ, et al. Coordination between the energy-consumption permit trading scheme and carbon emissions trading: Evidence from China[J]. Energy Economics, 2022, 116: 106433.

[37] KirikkaleliD, GüngörH, AdebayoTS. Consumption‐based carbon emissions, renewable energy consumption, financial development and economic growth in Chile[J]. Business Strategy and the Environment, 2022, 31(3): 1123–1137.

[38] MuhammadB, KhanS. Effect of bilateral FDI, energy consumption, CO2 emission and capital on economic growth of Asia countries[J]. Energy Reports, 2019, 5: 1305–1315.

[39] ZhouF, HuangZ, ZhangC. Carbon price forecasting based on CEEMDAN and LSTM[J]. Applied energy, 2022, 311: 118601.

The article "Analysis of China’s carbon market price fluctuation and international carbon credit financing mechanism using random forest model" was retracted in 2025. Reasons: concerns about the results or conclusions; concerns about the peer review; concerns about the authorship.

[40] SunW, HuangC. A carbon price prediction model based on secondary decomposition algorithm and optimized back propagation neural network[J]. Journal of Cleaner Production, 2020, 243: 118671.

[41] RazzaqA, SharifA, AnH, et al. Testing the directional predictability between carbon trading and sectoral stocks in China: New insights using cross-quantilogram and rolling window causality approaches[J]. Technological Forecasting and Social Change, 2022, 182: 121846.

